The article "Unraveling the probiotic efficiency of bacterium Pediococcus pentosaceus OBK05 isolated from buttermilk: An in vitro study for cholesterol assimilation potential and antibiotic resistance status" was published in 2021. Journal: PLoS One.

# Unraveling the probiotic efficiency of bacterium *Pediococcus pentosaceus* OBK05 isolated from buttermilk: An *in vitro* study for cholesterol assimilation potential and antibiotic resistance status

**DOI:** 10.1371/journal.pone.0259702

**Published:** 2021-11-04

**Authors:** Kiran Kumar Bhukya, Bhima Bhukya

**Affiliations:** Department of Microbiology, Centre for Microbial and Fermentation Technology, University College of Science, Osmania University, Hyderabad, Telangana, India; Government College University Faisalabad, PAKISTAN

## Abstract

The present study describes the probiotic potential and functional properties of the lactic acid bacterium *Pediococcus pentosaceus* OBK05 isolated from buttermilk. The isolate OBK05 was assessed for its probiotic properties. The isolate showed notable tolerance to pH 2.0 and 3.0 (8.44, 8.35 log CFU/mL), oxbile of 0.5% at 2 and 4 h of incubation (6.97, 6.35 log CFU/mL) and higher aggregation (auto-aggregation, adhesion to hydrocarbons) than the referral strain, *Lactobacillus acidophilus* MTCC 10307. The adhesion efficiency to HT-29 cells was found to be maximum, corresponding to 93.5% and 97% at 1 and 2 h incubation, respectively. In addition, the isolate OBK05 showed antagonistic solid activity against bacterial pathogens like *Pseudomonas aeruginosa* MTCC 424 and *Bacillus subtilis* MTCC 1133. The phenotypic antibiotic resistance of the isolate was examined before and after curing plasmids. Among the known five structural genes responsible for different antibiotic resistance, four genes indicating antibiotic resistance to kanamycin-*Aph* (3´´)-III, streptomycin-*strA*, vancomycin-*vanA* and ciprofloxacin-*gyrA* were detected by PCR amplification of genomic DNA. Further, the horizontal gene transfer from OBK05 isolate to pathogens was not found for these antibiotic resistance markers when filter and food mating were carried out as no transconjugants developed on media plates containing respective antibiotics. This indicates that the intrinsic resistance is harbored on chromosomal genes, and hence it is nontransferable to other microbes. In addition, strain OBK05 exhibited good DPPH scavenging activity of 56 to 77% and liberated free amino acid from conjugated bile acid. The strain OBK05 demonstrated a strong ability to reduce cholesterol at 12 h (17%), 24 h (27%) and 48 h (67%) of incubation.

## Introduction

One of the most common age-old indigenous fermented food products in India is naturally fermented buttermilk. The buttermilk is produced from pasteurized Indian bovine (cows/buffalo) milk fermented naturally in earthenware pots. The bacterial community in fermented buttermilk makes the final product nutritionally improved and safer to consume due to the production of bioactive compounds such as short chain fatty acids (Butyric acid, Lactic acid and Propionic acid), amino acids (Lysine, Arginine, Tyrosine and Tryptophan), vitamins (Vitamin B1, B6, and B12), enzymes like lipase, lactase and β-galactosidase [1]. The fermented buttermilk product also known as cultured milk product which a group of probiotic bacterial members ferments belong to the genera of *Lactococcus Lactis*, *Lactobacillus acidophilus*, *Leuconostoc mesenteroides subsp*. *mesenteroides*, *Bifidobacterium bifidum*, *Pediococcus pentosaceus*, *Bacillus cereus and Propionibacterium freudenreichii* [2].

Lactic acid bacteria (LAB) are catalase-negative, Gram-positive bacteria and consist of a wide range of genera, some of the important ones are, *Pediococcus acidilactici*, *Lactobacillus plantarum*, *Streptococcus thermophilus* and *Leuconostoc lactis* [3]. These microorganisms are the members of the gastrointestinal tract of animals, humans and are commonly found in dairy products such as fermented milk and cheese [4]. Microorganisms like *Pedioccocus* species which show antagonistic activity against gut pathogenic microflora, have been assessed and used as probiotics in functional foods [5].

Probiotics are non-pathogenic live microorganisms that exert health benefits when administered in sufficient amounts in the host [6]. These microorganisms are mainly associated with an improvement of bowel function, maintenance of gut microflora, modulation of lactose intolerance, diarrhoea prevention, lowering of hypertension, reduction of hypercholesterolemia, regulation of immune system and mitigation of specific allergies along with antimicrobial activity [6,7]. In fact, microflora imbalance in the digestive tract is considered one of the main factors in developing some malignancies and gastrointestinal diseases [8].

The selection of microorganisms as a good probiotic requires it to possess certain properties which include, stress tolerance (low pH, bile salts and body temperature), adhesion ability (aggregation and adhesion to intestinal epithelial cells), antipathogenic activity (production of antimicrobial metabolites and competing to pathogenic bacteria), safety (hemolytic activity, absence of virulence and nontransferable antibiotic resistant genes) and host-associated functional properties like, antioxidant, anti-cholesterol, anticancer, anti-obesity and secretion of functional molecules [9].

A LAB’s antibiotic resistance is an emerging food safety concern and the transfer of antibiotic resistance genes from potential probiotic bacteria to commensal or pathogenic microorganisms cannot be neglected. Therefore, antibiotic sensitivity profiling of probiotic bacterial strains intended for use as starter cultures is considered a significant part of safety [10]. Antibiotic resistance of bacteria can be either acquired or intrinsic. Acquired resistance is often identified as a resistance found only in certain members of a particular species, while intrinsic resistance is a native resistance present in all bacterial species. Inherent resistance is usually nontransferable to other bacterial species, and acquired resistance might be easily transferrable to other bacterial strains specifically if the resistance is located on plasmids [11]. In contrast, common susceptible microorganisms may acquire antibiotic resistance by developing new properties through mutations or acquire antibiotic resistance genes by conjugal gene transfer, mainly through the transmission of mobile genetic elements like transposons and plasmids. Bacteria use three independent mechanisms for gene transfer, namely, transformation, transduction and conjugation. Conjugation is an effective mechanism among these gene transfer mechanisms to transfer antibiotic resistant genes [12]. Moreover, probiotic *Lactobacillus* spp. isolated from fermented dry sausages harbored tetracycline-resistant gene *tet* (M) and transfer of antibiotic resistance was noted from *Lactobacillus* to *Enterococci* and *Lactococcus lactis* subsp. *lactis in vitro* indicating that *Lactobacillus* spp. were able to transfer the spread of antibiotic resistance gene [13].

The LAB strains may reduce the risk of oxidative damage by ion chelation, radical scavenging activity, enzyme inhibition, inhibition of ascorbate auto-oxidation and reduction activity [14]. Some probiotic strains produce extracellular polysaccharides like fructo-gluco oligosaccharide. Fructans and glucans exhibit antioxidant properties [15]. Probiotic microbial strains have the efficiency to transform bile salts through a bile salt de-conjugation mechanism [16].

The bile salt hydrolase (BSH) enzyme secreted by gut microbiota catalyzes the degradation of tauro-conjugated and glycol-conjugated bile acids through breakdown of amide bond and liberates free bile acids (chenodeoxycholic acid and cholic acid) and amino acids (taurine and glycine). Moreover, the BSH activity of gut microbiota is also involved in the metabolic reactions of mammals, including the control of cholesterol metabolism, inflammation, energy homeostasis and dietary lipid metabolism [17–19]. Unconjugated and conjugated bile salts are up taken in the gut by passive diffusion and absorbed by active transport in the ileum. Therefore, the BSH activity of probiotics is known to increase the de novo pathway of bile salts in the liver, leading to lowering serum cholesterol levels in the blood [20].

Cardiovascular disease is one of the major causes of death in developed countries. Reports suggest that, natural products and functional foods containing probiotics have been recommended as a beneficial dietary approach, which produces bioactive elements for lowering the total cholesterol and reducing the risk of heart disease [21]. Therefore, considerable attention is being paid to the useful effects of probiotic strains of fermented milk products on human lipid metabolism. Numerous studies have suggested a moderate cholesterol-reducing action of food products that have been supplemented with some strains of probiotic organisms in humans [22].

Therefore, the objectives of the present study were to investigate the ability of *Pediococcus pentosaceus* OBK05 strain, isolated from buttermilk, to tolerate hostile conditions of the intestine such as acid, bile and other properties like antibacterial as well as antibiotic resistance status whether located on chromosome or plasmid, cell adhesion property, antioxidant activity and cholesterol-lowering ability.

## Materials and methods

### Buttermilk

Buttermilk is a popular naturally fermented milk product prepared by rural communities from pasteurized/heat-treated bovine (cow’s) milk which is allowed to ferment naturally in an earthenware pot for one to two days at a suitable temperature to form a thick curd. The microbial content liable for the fermentation is derived from either water, air, raw milk or walls of the earthenware pot. The curdled thick milk is then mixed with equal amount of water and churned to make buttermilk.

### Sample collection and processing

A total of ten buttermilk samples were collected in sterile polythene bags from rural households of Warangal, Khammam and Nalgonda districts of Telangana state, India and brought to the laboratory in an icebox at 4°C. Tenfold serial dilutions were prepared with one mL of each sample to get well-isolated colonies of lactic acid bacteria when inoculated on MRS agar medium plates.

### Isolation and growth conditions

Diluted samples were inoculated on de Man, Rogosa and Sharpe (MRS) agar medium (Himedia, India) with 1% CaCO_3_ and incubated at 37°C for 2 days to distinguish acid-producing bacteria from others. The sugar fermentation ability of all the isolates was performed using 1% (w/v) sugar in MRS broth. Glucose, fructose, sucrose, galactose, maltose, xylose, arabinose, mannose, trehalose, lactose, raffinose, ribose and mannitol were used in this test and incubated at 37°C for 24 h. After incubation, the sugar fermentation pattern was observed by the addition of Andrade’s indicator to all the tubes where the pink colour tube indicates positive for sugar fermentation [15].

### *In vitro* probiotic characteristics

#### Tolerance to low pH and bile

The acid and bile tolerance ability of microbial isolates was assessed according to the previous method described [23]. Acid tolerance of microbial strains was assessed in sterile saline with pH adjusted to 2.0, 3.0, and 4.0 and incubated for 0, 2 and 4 h. Bile tolerance of isolates was assessed with 0.5% ox-bile (Himedia, India) and incubated for 0, 2 and 4 h at 37°C. After incubation, the cell viability (log CFU/mL) was observed by culturing on MRS agar. The *Lactobacillus acidophilus* (MTCC 10307) is used as a positive control for both experiments.

#### Molecular characterization

The selected isolate was characterized by sequencing its 16S rRNA (Macrogen, South Korea). The obtained partial sequence was compared with the database sequences by BLAST search engine in the nucleotide database of National Centre for Biotechnology Information (NCBI) for similarity. The 16S rRNA gene sequence of the isolate was deposited in the GenBank database. Phylogenetic tree was constructed by UPGMA method using MEGA 7.0 software for the relatedness of the isolate with the database strains.

#### Auto aggregation

The aggregation ability of the isolates was studied according to the previous method described [24]. The percentage of auto-aggregation was expressed as:

$$\%=1‐A_{t}/A_{0}\;X\;100$$

Where A_t_ is the absorbance at 6, 12, 24 h and A_0_ is the absorbance at 0 h.

#### Bacterial adhesion to hydrocarbon (BATH)

Bacterial adhesion to hydrocarbon (Cell surface hydrophobicity) was carried out according to a previous protocol [25]. The percentage of bacterial hydrophobicity (H%) was calculated using the following formula.


$$H\%=(1–A_{1}/A_{0})\;X\;100.$$

Where, A_1_ is the absorbance of an aqueous phase, and A_0_ is the initial absorbance.

### Adhesion to intestinal epithelial cells

#### Maintenance and propagation of cell lines

The human intestinal epithelial cell line HT-29 (Colon adenocarcinoma cells) was procured from National Center for Cell Science (NCCS), Pune, India, and maintained in Dulbecco’s Modified Eagle’s Medium (DMEM) with 10% (v/v) heat-inactivated filtered Fetal Bovine Serum (FBS) and Antibiotic-Antimycotic solution (100X, Thermo fisher scientific, USA). Cells were cultured in 25 cm^2^ tissue culture flasks at 37°C by humidifying with 5% CO_2_ and 95% air in a CO_2_ incubator (New Brunswick, Galaxy 170S, Germany) for further experiments.

#### Preparation of CFDA-SE dye and bacterial labelling

According to the method described [26], the stock solution was prepared by dissolving 10 mg/mL of carboxyfluorescein diacetate succinimidyl ester (CFDA-SE) in DMSO and further diluted in 5.9 mL of ethanol to 1.7 mg/mL concentration and stored at -20°C. Further, a working solution was prepared by adding 1mL of stock solution to 140 mL of PBS to give 2 μM final attention for bacterial labelling. Bacterial labelling was carried out according to the previous method described [8].

#### Cell adhesion assay by flow cytometry

The interaction between HT-29 cells and bacterial cells was analyzed by flow cytometry (BD FACS Aria II—BD Bio Science, San Jose, USA). Data represented on both scattered plot and histogram plots were analyzed by CELL Quest software (Becton Dickinson). A sample of auto-fluorescent HT-29 cells was initially loaded and a gate was created in the histogram based on the most number of cells that were spotted on the forward-scattered light (FSC) and side-scattered light (SSC). An amount of 1mL epithelial cells was added to 0.5 mL of labelled bacterial suspension in each of the sterile 15 mL falcon tubes and incubated at 37°C for 1 h and 2 h by placing the tubes in the end over end rotation. Before the adhesion assay, the cells were fixed with 37% formaldehyde and observed for adhesion based on the mean fluorescence intensity (MFI). The percentage of adhesion was calculated based on the ratio of MFI at 1 h and 2 h. Unstained HT-29 cells and bacterial suspension were treated as control, while stained HT-29 and bacterial suspension were treated as test samples.

Adhesive efficiency of the bacterial isolate to HT-29 epithelial cells was carried out in a six-well tissue culture plate [27]. After attaining 60% confluency, cells were inoculated with a known concentration of bacterial cells (10^8^) and incubated at 37°C for 2 h. After incubation, the number of adhesive bacterial cells were counted randomly under an inverted microscope (EVOS M 5000, Thermo fisher scientific) in 20 microscopic fields and reported as non-adhesive (<40 bacteria), adhesive (40–100 bacteria) and strongly adhesive (>100 bacteria).

#### Haemolytic and DNase activity

The haemolysis of the LAB isolate was observed using the Columbia blood agar (Himedia, India) plates containing 1% blood (from human volunteers) and incubated at 37°C for 24 h and observed for haemolytic (γ-non-haemolytic, α and β-haemolytic) activity [28]. The bacterial DNase (Deoxyribonuclease) activity was analyzed by inoculating the culture of LAB isolate on the surface of the DNase test agar medium (HiMedia). A clear pink, purple zone around the bacterial colonies was considered positive for DNase activity [28].

#### Antagonistic activity against bacterial pathogens

The antagonistic activity of LAB cell free-supernatant (CFS) against bacterial pathogens was performed using the agar-well diffusion method [29–31]. Indicator microorganisms like *Bacillus subtilis* MTCC 1133, *Escherichia coli* MTCC 452, *Klebsiella pneumoniae* MTCC 4031, *Pseudomonas aeruginosa* MTCC 424, *Salmonella typhi*, *Staphylococcus* aureus MTCC 3160, *Lactobacillus acidophilus* MTCC 10307 and *Saccharomyces cerevisiae* were incubated in Tryptic Soy Broth, MRS and YEPD broth for 24 h, diluted until an O.D_600_ of 0.05 was attained, then spread on respective agar medium as mentioned above. The CFS of LAB was prepared by centrifugation of overnight culture of LAB isolate at 10,000 rpm/10 min at 4°C, and the pH of the supernatant was adjusted to 6.5 ± 0.2 using 2 M NaOH. Subsequently, 50 μl of CFS of LAB isolate was placed in each agar-well and incubated at 37°C for 24 h to determine the zone of inhibition around the wells.

#### Determination of antibiotic sensitivity and status of antibiotic resistance

The antibiotic sensitivity of the LAB isolate was determined on MRS agar plates using the single disc diffusion method [32]. Antibiotic discs for Amoxicillin (10μg/disc), Ampicillin (10μg/disc), Gentamicin (10μg/disc), Kanamycin (05μg/disc), Streptomycin (25μg/disc), Erythromycin (15μg/disc), Vancomycin (10μg/disc), Ciprofloxacin (05μg/disc), Norfloxacin (10μg/disc), Clindamycin (10μg/disc), Lincomycin (10μg/disc), Polymixin B (300μg/disc), Tetracycline (10μg/disc), Trimethoprim (10μg/disc) and Rifampicin (05μg/disc) were used. The sensitivity and resistance of the isolates were determined by the formation of a clear zone around the discs, and the antibiotic resistance status of lactic acid bacteria was assessed to know whether it is a plasmid or chromosomal borne.

#### Plasmid curing

Plasmids of LAB isolate were cured to assess the antibiotic resistance status as previously described [11]. Before curing the plasmids, protoplasts were prepared by centrifuging overnight grown culture of LAB isolate (O.D_600_ of 0.5 to 1.0) at 10000 rpm for 5min and washed twice with 10 ml of milli-Q water, re-centrifuged, and re-suspended in 5 ml protoplast buffer (0.5 M sucrose, 20 mM MgCl_2,_ 0.2 M sodium phosphate, pH 7.0). Subsequently, cells were added with an equal volume of 10 mg/ml lysozyme (Sigma-Aldrich, Inc.) and incubated at 37°C for 1 h for lysis of protoplasts. The protoplasts were harvested by centrifugation at 3000 X g for 15min, re-suspended in 2 ml protoplast buffer and serially diluted for regeneration. Sample from higher dilution was then inoculated on MRS agar medium with 0.5 M sucrose for regeneration. Antibiotic sensitivity of regenerated plasmid-cured protoplasts was identified on MRS agar plates with different antibiotics.

#### Plasmid isolation

Plasmid DNA was extracted from LAB isolate before and after curing the plasmids to confirm the efficiency of curing, as previously reported [11]. In brief, the bacterial cells (1.5 mL) were harvested in microcentrifuge tubes by centrifugation at 2000 rpm for 2 min, and plasmid DNA was extracted using MiniKit (Qiagen, USA) according to the manufacturer’s instructions. The extracted plasmid DNA was observed by agarose gel electrophoresis.

#### Detection of antibiotic resistance genes

Extraction of genomic DNA from overnight LAB culture was carried out with the Xpress DNA kit (MagGenome Technologies Pvt. Ltd., India), according to the manufacturer’s instructions. The existence of genes associated with resistance to antibiotics in the LAB strains was determined by Polymerase chain reaction (PCR) amplification using the specific primers for known antibiotic resistance genes and conditions. The PCR amplification was carried out in a thermal cycler A48141 (Applied biosystems, Germany) using the following program: Initial denaturation at 94°C for 3 min, 35 cycles of 94°C for 1min, annealing temperature for the specific primer and 72°C for 1 min, and final extension step of 72°C for 7 min. The amplified PCR DNA template (5μl) was separated by gel electrophoresis on 1% agarose (w/v) gel.

### Transfer of antibiotic resistance

#### Filter mating

Transfer of antibiotic-resistant genes from LAB isolates to pathogenic microorganisms was examined by the filter mating method [13]. For this, LAB isolate (donor) and intestinal pathogen (recipient) were grown separately in a non-selective medium up to the mid-exponential phase of growth (~ 4h). The donor cells and the recipient cells were mixed in 1:1 ratio, and the mixture was filtered through a sterile composite cellulose ester filter (0.45μm, HAWP-02500, Millipore) using a swinex filter holder (SX 02500, Millipore). After filtration, sterile peptone physiological saline solution (PPS- 8.5gm/L NaCl and1gm/L peptone) was passed through the filters to trap the cells more tightly into the membrane. The filters were placed on a non-selective agar medium and incubated at recipient bacterial growth conditions. After incubation, filters were washed with 2ml PPS solution, filtrates (mating mixture) were spread on selective antibiotic agar medium plates and incubated at 37°C for 24–48 h, to screen for antibiotic-resistant transconjugants.

#### Food mating

A food mating experiment was carried out in a biosafety cabinet as previously described [12]. Cheese slices (4cm x 3cm) were placed in sterile petri dishes inoculated with mixed strains of LAB isolate (donor) and intestinal pathogen (recipient) in a 1:1 ratio and incubated at 37°C for 24 h. After incubation, the cheese pieces were washed with 2 mL sterile PPS solution and screened for transconjugants.

#### Confirmation of transconjugants

The obtained transconjugants from mating experiments were grown in selective broth without antibiotics before being spread onto agar medium petri dishes containing antibiotics. The transfer of antibiotic resistance marker was examined based on the antibiotic sensitivity pattern using Kirby-Bauer disc diffusion method.

### Screening for functional properties

#### Antioxidant activity

Antioxidant activity of bacterial cell-free supernatant (CFS) was investigated according to the previous method described [33]. The antioxidant activity was quantified by the following formula:

$$DPPH\;activity\;(\%)=(ABS_{C}‐ABS_{S})/S\;X\;100.$$

Where ABS_C_ and ABS_S_ are the absorbance of the control and test samples, respectively. S is the volume (mL) of a sample.


HRSactivity(%)=(As–Ac)/(Ab–Ac)X100

Where A_S_ is the absorbance of sample, A_C_ is the absorbance of the control (deionized water), and A_b_ is the absorbance of the solution without sample and H_2_O_2._

#### Bile salt hydrolase (BSH) activity

The bile salt hydrolase (BSH) activity of LAB isolate was determined by analyzing free amino acids liberated from conjugated bile salt by LAB isolate [34]. The BSH activity was determined using sodium taurocholate (0.5% w/v). The formation of a halo around the colonies indicates BSH activity. MRS agar plate without sodium taurocholate was treated as a negative control.

#### Cholesterol assimilation ability

The cholesterol stock solution of 1 g/L (w/v) was prepared by dissolving in 20% isopropanol and tween 80 in a volumetric flask. The working solution was design from the stock to obtain aliquots of 1mg/mL and then added to the medium. The test medium, sterile MRS broth supplemented with 1 mg/mL (v/v) cholesterol, was inoculated with an overnight culture of LAB isolate (1% v/v, 10^6^ CFU/mL) and incubated at 37°C for 12, 24 and 48 h. After incubation, bacterial cells were separated by centrifugation (10000 X g, 10 min, 4°C), and the spent broth, along with un-inoculated sterile broth was analyzed for their cholesterol content. Cholesterol content was analyzed on High-pressure liquid chromatography (HPLC, Shimadzu, Japan) as previously described [35], which is equipped with a variable wavelength detector and shim-pack GIST C18 column (250 X 4.6mmI.D., 5μm, Phenomenex, USA). Isopropanol and acetonitrile (50:50 v/v, HPLC-grade, Merck, India) were used as mobile phase, and 1mL/min isocratic elution was performed with column temperature of 30°C by injecting 20 μl of the sample. Cholesterol in samples was detected at 254 nm and 5 min retention time.

### Statistical analyses

Sigma Plot 12.5 was used for statistical data analysis. Each experiment was carried out in triplicate, and data was expressed as mean value ± standard deviation, and the mean value of each experiment was analyzed by two way ANOVA with the value of *P* <0.05 was considered as significant.

## Results and discussion

### Isolation and identification

A total of thirty lactic acid bacterial (LAB) isolates (OBK 01 to OBK 30) were isolated from buttermilk using an MRS medium supplemented with calcium carbonate (CaCO_3_). Calcium carbonate is used to distinguish acid-producing bacteria from others. Differentially expressed colonies with a clear zone of hydrolysis were selected as LAB isolates. An analysis of utilization pattern of 13 sugars by LAB isolates showed that all the isolates could utilize galactose, glucose, fructose, sucrose and maltose but for remaining carbohydrates, organisms showed different utilization pattern. The carbohydrate utilization efficiency of LAB isolates depends on their fermentation habitat, natural mutations and physiological conditions [15]. Based on the carbohydrate utilization efficiency of OBK04, OBK05, OBK08 and OBK12, the isolates which fermented lactose and showed positive β-galactosidase activity were selected for further studies.

### Acid and bile tolerance

The most important step for selecting probiotic LAB isolates is their ability to survive under hostile intestine conditions like high bile concentration (in small intestine) and low pH (gastric condition) for successful passage through the gastro intestinal tract to the large intestine. All the four isolates were found to tolerate low pH of 2.0 and 3.0 with various survival rates after incubation for 4 h (Table 1). The viable count of OBK05 was significantly (*p* <0.05) higher than those of the other three isolates OBK04, OBK08, and OBK12 at pH 2.0 and 3.0. However, *L*. *acidophilus* MTCC10307, the standard/reference organism, showed the viability of only 8.45 and 8.40 CFU/mL at pH 2.0 and 3.0, respectively. Previous studies reported lower survivability of various probiotic strains in acidic conditions. The probiotic organism, *P*. *pentosaceus* VJ35 showed 7.12, and 7.57 CFU/mL [36], and *P*. *pentosaceus* OF31 showed 7.95 and 8.08 CFU/mL [37] tolerance after 4 h of incubation at pH 2.0 and 3.0 respectively.

**Table 1:** Acid tolerance ability of Lactic acid bacterial (LAB) isolates.

Growth in log CFU/mL at different time intervals				
Isolates	pH	0h	2h	4h
OBK04	pH 2.0	9.53 ± 0.23*	9.45 ± 0.15*	9.35 ± 0.43**
	pH 3.0	9.25 ± 0.12	9.12 ± 0.51	8.98 ± 0.37
	pH 7.0	9.27 ± 0.15	9.35 ± 0.50	9.51 ± 0.35
OBK05	pH 2.0	9.12 ± 0.35	8.97 ± 0.47	8.44 ± 0.43**
	pH 3.0	9.20 ± 0.12	8.80 ± 0.27	8.35 ± 0.26***
	pH 7.0	9.15 ± 0.13	9.10 ± 0.25	9.42 ± 0.37
OBK08	pH 2.0	9.15 ± 0.35	8.77 ± 0.37	8.57 ± 0.37*
	pH 3.0	8.87 ± 0.44	8.68 ± 0.33	8.14 ± 0.27****
	pH 7.0	9.05 ± 0.14	9.12 ± 0.18	9.37 ± 0.41
OBK12	pH 2.0	9.21 ± 0.35	9.06 ± 0.35	8.25 ± 0.18****
	pH 3.0	9.30 ± 0.28	8.90 ± 0.11	8.65 ± 0.25*
	pH 7.0	9.20 ± 0.11	9.25 ± 0.37	9.41 ± 0.37
*L*. *acidophilus*	pH 2.0	9.20 ± 0.10	9.01 ± 0.15	8.45 ± 0.37**
	pH 3.0	9.05 ± 0.17	8.87 ± 0.47	8.40 ± 0.67**
	pH 7.0	9.21 ± 0.37	9.17 ± 0.27	9.37 ± 0.38

The experiments were carried out in triplicates (mean ± standard deviation). Statistical difference was determined by Tukey’s multiple comparison test.

*p ≤ 0.05

**p ≤ 0.01

***p ≤ 0.001

****p ≤ 0.0001.

Tolerance to bile is one of the essential attributes of probiotics, as high concentrations of bile salts are known to be toxic to the bacterial cells and affect cell viability [23]. All the four isolates including standard probiotic strain resisted 0.5% ox-bile, while, OBK05 showed a significant (*p* <0.05) difference in tolerance (6.97 and 6.35 CFU/mL) with other isolates at 2 and 4 h (Table 2). The obtained results are in accordance with previous studies where the probiotic strains isolated from rumen liquor showed similar viability [38], and *Lactobacillus* strains isolated from kimchi showed similar viability in bile salts [39]. The obtained results suggested OBK05 as the most promising strain to tolerate low pH and high bile concentration compared to other LAB isolates. Therefore, the isolate OBK05 was selected for further studies.

**Table 2:** Tolerance of Lactic acid bacterial (LAB) isolates to Ox bile.

Growth in log CFU/mL at different time intervals				
Isolates	Bile (%)	0h	2h	4h
OBK04	0.0	8.18 ± 0.51	8.30 ± 0.27	8.44 ± 0.34
	0.5	7.98 ± 0.44	6.93 ± 0.32****	6.26 ± 0.44****
OBK05	0.0	7.86 ± 0.41	7.96 ± 0.44	8.05 ± 0.26
	0.5	7.43 ± 0.47	6.97 ± 0.47**	6.35 ± 0.41****
OBK08	0.0	8.25 ± 0.72	8.51 ± 0.39	9.32 ± 0.24
	0.5	7.95 ± 0.36	7.68 ± 0.46*	7.61 ± 0.62****
OBK12	0.0	7.20 ± 0.14	7.38 ± 0.42	7.86 ± 0.52
	0.5	7.22 ± 0.27	6.67 ± 0.25	6.60 ± 0.62***
*L*. *acidophilus*	0.0	8.05 ± 0.17	8.12 ± 0.11	8.20 ± 0.25
	0.5	7.90 ± 0.23	6.35 ± 0.33****	6.15 ± 0.37****

The experiments were carried out in triplicates (mean ± standard deviation). Statistical difference was determined by Tukey’s multiple comparison test.

*p ≤ 0.05

**p ≤ 0.01

***p ≤ 0.001

****p ≤ 0.0001.

### Molecular characterization

The selected LAB isolate was characterized based on a 16S rRNA sequence. NCBI database showed that the 16S rRNA gene sequence of OBK05 (Gene bank accession number MF996786; 1598bp) matches 100% with *Pediococcus pentosaceus* type strain Ni1379 and <100% with other *Pediococcus* species. Based on similarity results, the LAB isolate OBK05 was identified as *Pediococcus pentosaceus* OBK05. The phylogenetic tree was constructed for complete 16S rRNA gene sequence of LAB isolate OBK05 by UPGAMA method using MEGA7.0 software which showed the relative position of *P*. *pentosaceus* OBK05 with *P*. *pentosaceus* Ni1379 with 1000 bootstrap replicates (Fig 1).

**Fig 1:** Phylogenetic tree representing the relationship of OBK05 with other members of *Pediococcus* spp.

### Auto-aggregation and hydrophobicity

Aggregation between bacterial cells of the same strain (auto-aggregation) is important in many ecological niches, specifically in humans as it increases the possibility of bacterial balance in the gastrointestinal tract [5]. Additionally, colonization of probiotic microorganisms in the gastrointestinal tract improves host defense and prevents the entry of external human pathogens [40]. Auto-aggregation is an essential property of probiotic strains for adhesion to human intestinal epithelial cells [38]. Auto-aggregation ability of OBK05 strain was measured after 6, 12 and 24 h of incubation (Fig 2A). The obtained values differed greatly with the incubation period and were firmly strain-dependent (*p* < 0.05). Strain OBK05 aggregated quickly with 60% aggregation ability during the first 6 h, and after 24 h of incubation, the aggregation ability increased to 87%. The auto-aggregation ability of OBK05 was significantly (*p* <0.05) greater than that of the standard probiotic strain *L*. *acidophilus* (70%) after 24 h, indicating its high efficiency of aggregation compared to the standard probiotic strain. The present results are in accordance with previous studies where *P*. *pentosaceus* D56 strain isolated from jeotgal showed autoaggregation of 69% after 24 h incubation [41]. Similarly, *P*. *pentosaceus* Wikim86 strain isolated from kimchi showed 85% aggregation after 24 h incubation [1].

**Fig 2:** Aggregation ability of *P*. *pentosaceus* OBK05 and *L*. *acidophilus*. (A) Auto- aggregation ability (B) Cell surface hydrophobicity. Experiments were carried out in triplicates, and data with Error bars representing the Mean ± S.D. values of the independent investigation (p<0.05).

The hydrophobicity of OBK05 strain for xylene and chloroform was found to be 88% and 81%, respectively (Fig 2B) while, the hydrophobicity of standard probiotic *L*. *acidophilus* strain for chloroform and xylene was 74% and 78%, respectively. This indicates that the isolate has higher hydrophobicity and a strong electron donor profile. Our values are higher than the previous reports where *P*. *pentosaceus* MZF16 strain isolated from dried ossban exhibited 61% [42] and *P*. *pentosaceus* D56 strain showed 33% hydrophobicity to xylene [41]. Similarly, a previous study revealed that *P*. *pentosaceus* OZF strain isolated from human breast milk exhibited 42% affinity to chloroform [43]. Lower hydrophobicity is firmly linked to polysaccharide and higher hydrophobicity is associated with glycoproteins on the surface of bacteria [42].

### Adherence assay

Flow cytometry is one of the most accurate techniques used for assessing the adhesion of bacterial cells to intestinal epithelial cells and therefore was used in the present study [44]. The adhesion efficiency of *P*. *pentosaceus* OBK05 strain to human intestinal epithelial cells (HT-29) was examined by flow cytometry after staining the live bacterial cells with CFDA-SE. A shift in fluorescence intensity (FLI) indicates adhered microbial cells to HT-29 cells (Fig 3). The FLI peak was near the y-axis indicating no adhesion between OBK05 and intestinal epithelial cells at 0 h (Fig 3A). The adhesion efficiency of fluorescently-labeled OBK05 strain with HT-29 cells was observed as 93.5%, and 97% at 1 and 2 h, respectively, as the peaks on FLI were near the x-axis due to solid adhesion between OBK05 and HT-29 cells (Fig 3B and 3C). Further to support the findings of adhesion efficiency, six-well tissue culture plate count was carried out. The counts of ˃100 bacteria are considered strongly adhesive, and >100 bacteria were found at 1 and 2 h treatments but not at 0 h. A previous study revealed that *L*. *plantarum* DF9 isolated from indigenous food sources showed 29.94% adhesion [26].

**Fig 3:** Adhesion efficiency of *P*. *pentosaceus* OBK05 by flow cytometry. (A) HT-29 cells co-incubated with CFDA-labeled OBK05 at 0 h, (B) HT-29 cells co-incubated with CFDA-labeled OBK05 for 1 h and (C) HT-29 cells co-incubated with CFDA-labeled OBK05 for 2 h. Arrows indicate that the adhesion of live OBK05 strain was stained with Giemsa dye on HT-29 cells for 1 and 2 h and showed ˃100 bacterial counts respectively.

### Haemolytic and DNase activity

The haemolytic and DNase activities of microorganisms are crucial markers for their pathogenic nature. The isolate OBK05 displayed no hemolytic activity (γ-haemolysis) when tested on a blood agar medium. The same results have been previously obtained with *P*. *pentosaceus* MZF16, a dried ossban probiotic [42]. An investigation [15] revealed that, *P*. *pentosaceus* SW01 strain has the ability of α-haemolysis which contrasts with the present results. The DNase enzyme activity was not found with OBK05 strain as there was no pink colour formation around the colonies on the DNase test agar medium indicating that it is non-pathogenic and considered safe for human probiotic applications.

### Antagonistic activity

The antagonistic activity of probiotic organisms comprises the production of antibacterial compounds, including organic acids, free fatty acids (FFAs), hydrogen peroxide and low molecular weight compounds called bacteriocins [37,42]. The isolate *P*. *pentosaceus* OBK05 effectively inhibited the growth of six bacterial pathogens like *Bacillus subtilis* MTCC 1133, *E*.*coli* MTCC 452, *Klebsiella pneumoniae* MTCC 4031, *Pseudomonas aeruginosa* MTCC 424, *Salmonella typhi* and *Staphylococcus aureus* MTCC 3160 with inhibition zones of 9.5, 9.1, 8.5, 10.0, 9.0 and 9.0 mm, respectively. Incontrast, the isolate did not show any effect on standard probiotic organisms like *Lactobacillus acidophilus* MTCC 10307 and *Saccharomyces cerevisiae* MTCC 25158 (Fig 4A–4H). These results indicated that *P*. *pentosaceus* OBK05 is a strong growth inhibitor of *Bacillus subtilis* and *Pseudomonas aeruginosa*, which are important opportunistic human pathogens [45]. Similarly, a broad spectrum of antagonistic activity observed among *Pediococcus* and *Lactobacillus* species have been reported [46,47]. Foodborne illness can occur with contaminated food or pathogens established in the human digestive system, producing toxins that lead to diarrhea, aches, vomiting and fever, etc. Therefore, probiotic diversity in the human gut prevents colonization by pathogens via competition by nutrition and production of antibiotic-related secondary metabolites. Further, the antimicrobial activity exhibited by these probiotic microorganisms may be helpful to control the unwanted pathogenic microorganism either in the gastrointestinal tract or in foods [45].

**Fig 4:** Antagonistic activity of *P*. *pentosaceus* OBK05 against human pathogens. (A) *Bacillus subtilis*, (B) *E*.*coli*, (C) *Klebsiella pneumoniae*, (D) *Pseudomonas aeruginosa*, (E) *Salmonella typhi*, (F) *Staphylococcus aureus*, (G) *Lactobacillus acidophilus* and (H) *Saccharomyces cerevisiae*. Arrows indicate the effect of OBK05 isolate on pathogens in the form of zone of inhibition (mm) around the wells. Experiments were performed in triplicates, and Data represented as the means ± S.D. of three independent experiments.

### Screening for antibiotic resistance

Probiotic LAB are generally recognized as safe. However, due to their excessive consumption, the safety of these probiotic organisms is becoming a prerequisite, with antibiotic resistance as a prominent issue [10]. Prior to plasmid curing, the strain OBK05 was resistant to antibiotics like kanamycin, streptomycin, vancomycin, ciprofloxacin, norfloxacin, and trimethoprim and exhibited susceptibility to amoxicillin, ampicillin, gentamicin, erythromycin, clindamycin, lincomycin, tetracycline and rifampicin. Similar results were observed for *P*. *pentosaceus* CRAG3 isolated from fermented cucumber [48]. After successful curing of OBK05 plasmid, the strain showed resistance to same antibiotics like kanamycin, streptomycin, vancomycin, ciprofloxacin, and norfloxacin, indicating that the resistance is harboured on chromosomal genes and only for the trimethoprim antibiotic, the strain showed susceptibility after plasmid curing, indicating that the resistance is plasmid-borne (Table 3). Plasmid band (10000 bp) was found on agarose gel before curing the plasmids but not after curing the plasmids, clearly indicating that plasmids were efficiently cured of the bacterial cells (Fig 5).

**Fig 5:** Detection of *P*. *pentosaceus* OBK05 plasmid DNA before and after plasmid curing. From left to right Lane (M): 1 kb DNA marker, Lane 1: Plasmid before curing, Lane 2: Plasmid after curing.

**Table 3:** Antibiotic sensitivity of *P*. *pentosaceus* OBK05 using different antibiotic discs before and after plasmid curing.

Group	Antibiotic	Concentration (μg)	Sensitivity before plasmid curing	Sensitivity after plasmid curing
β- lactam	Amoxicillin (AMX)	10	S	S
	Ampicillin (AMP/AX)	10	S	S
Aminoglycosides	Gentamicin (GEN)	10	S	S
	Kanamycin (K)	05	R	R
	Streptomycin (S)	25	R	R
Macrolides	Erythromycin (E)	15	S	S
Glycopeptides	Vancomycin (VA)	10	R	R
Fluoroquinolone	Ciprofloxacin (CIP)	05	R	R
	Norfloxacin (NX)	10	R	R
Lincosamides	Clindamycin (CD)	10	S	S
	Lincomycin (L)	10	S	S
Tetracyclin	Tetracyclin (TE)	10	S	S
Trimethoprim	Trimethoprim (TR)	10	R	S
Rifampicin	Rifampicin (RIF)	05	S	S

Zone of inhibition of microbial growth: R-resistant (0–2 mm); S-susceptible (3 – 10mm).

### Detection of antibiotic resistance genes

The genetic determinant responsible for the phenotypic antibiotic resistance was observed in the strain OBK05. The presence of known structural genes related to antibiotic resistance like kanamycin-*Aph* (3´´)-III, streptomycin-*strA*, vancomycin-*vanA* and ciprofloxacin-*gyrA* were examined by PCR amplification followed by determining the size of the amplicons. Though the PCR was not carried out to know the genetic basis of norfloxacin resistant genes, the strain showed resistance to the norfloxacin antibiotic. The genetic basis for the rest of the four antibiotic resistance genes was found by PCR amplification and found to be chromosomal located and, hence, nontransferable (Table 4).

**Table 4:** Primers used for detection of antibiotic resistance genes of *P*. *pentosaceus* OBK05.

Antibiotic resistance	Resistance gene	Primers (5’ to 3’)	Annealing temperature (°C)	References
Kanamycin	Aph (3´´)-III	F-5’-GCCGATGTGGATTGCGAAAA-3’	52	Ouoba et al., 2008
		R-5’-GCTTGATCCCCAGTAAGTCA-3’		
Streptomycin	strA	F-5’-CTTGGTGATAACGGCAATTC-3’	55	Ouoba et al., 2008
		R-5’-CCAATCGCAGATAGAAGGC-3’		
Vancomycin	vanA	F-5’-AACAACTTACGCGGCACT-3’	55	Ouoba et al., 2008
		R-5’-AAAGTGCGAAAAACCTTGC-3’		
Ciprofloxacin	gyrA	F-5’-GAYTATGCWATGTCAGTTATTGT-3’	45	Ouoba et al., 2008
		R-5’-GGAATRTTRGAYGTCATACCAAC-3’		
Norfloxacin	-	-	-	-

### Detection of antibiotic resistance gene transfer by filter and food mating methods

The filter mating method was used to examine the conjugal transferability of antibiotic resistance. The LAB strain OBK05 that is resistant to most antibiotics was taken as donor and antibiotic susceptible food pathogens like *Enterococcus faecalis*, *Staphylococcus aureus*, *Klebsiella pneumoniae* and *Escherichia coli* were taken as recipients. Prior to the curing plasmid, the strain OBK05 was conjugally mated with the above recipients by filter mating. Only for trimethoprim (TR) antibiotic, the resistance was successfully transferred to the recipients, at a frequency of 2X10^4^, 10^6^, 2X10^5^ and 3X10^4^ transconjugants per recipient and tested to confirm that the obtained isolates were true conjugants and do not reverse mutate again. There were no transconjugants obtained with kanamycin-*Aph* (3´´)-III, streptomycin-*strA*, *vancomycin-vanA* and norfloxacin antibiotics which revealed the presence of nontransferable chromosomal borne antibiotic resistance in the LAB strain OBK05. Earlier studies reported *in vitro* transfer of *tet*(M), *erm*(B) and *tet*(S) antibiotic resistance from different LAB strains such as *Lactobacillus plantarum*, *Lactobacillus alimentarius*, *Lactobacillus reuteri and Lactococcus lactis* to *Lactobacillus* and *Enterococci* spp. at frequencies ranging between 4.4X10^8^ to 4.5X10^10^ [13,36,49]. According to previous studies [49], the African isolate *L*. *reuteri* 12002 carrying *erm* (B) resistance gene is transferable to other microorganisms and not safe to be used as a probiotic but can be used for meat preservation. However, till now, no successful conjugal transfer has been reported for *pediococcus* spp.

Mating experiments were also conducted in food matrices using the same donor and the recipient organisms as in the filter mating method. The mating trial was carried out on the surface of the cheese. The successful presumptive transconjugants were obtained before plasmid curing for trimethoprim (TR) antibiotic with an effective conjugation frequency of around 2.5X10^4^, 2X10^6^, 3X10^5^ and 3.4X10^4^ per recipient, which was slightly higher than the values of the filter mating method and is in accordance with previous study [12]. After successful curing of plasmid, no transconjugants were found. The antibiotic sensitivity of each donor, recipient and transconjugants were observed using Kirby-bauer disc diffusion method. In addition, it was observed that the strain OBK05 carrying chromosomal borne antibiotic resistance did not lose its probiotic properties for several generations. This organism with probiotic properties might be beneficial for weakening the infections, treating contagious diseases, and rebalancing the normal gut microflora when used along with strong antibiotics [11,32].

### Free radical scavenging ability

The antioxidant activity of probiotic strain OBK05 is expressed in the form of scavenging of DPPH and HRS. The OBK05 strain showed >56.15% DPPH scavenging activity at lower concentrations (1:1) of cell-free supernatant (CFS). Increased antioxidant activity (60.6 to 77.83%) (p <0.05) was observed with the increase in the concentration of CFS (1:2 to 1:5). The HRS activity was reduced to 25.64% at a lower concentration of CFS and was increased (42.4%) with the increased concentration of CFS (1:5). The CFS showed weaker HRS activity than that of the DPPH scavenging activity (p <0.05). However, the antioxidant activity of CFS was higher than that of the MRS broth (negative control) in scavenging the HRS and DPPH radicals. The CFS showed lower DPPH and HRS activity than ascorbic acid (93.43 and 81.63%), the positive control (p <0.05) (Fig 6). These results reveal that OBK05 can be considered a probiotic bacterium with great antioxidant potential to reduce the free radicals in food and feeds. The obtained values are higher than the previous reports where the probiotic *P*. *pentosaceus* Wikim 85 and Wikim 86 showed 32% and 29% antioxidant activity, respectively [39]. The present findings are in agreement with [33] and [3]. The radical scavenging activity may be due to the secretion of secondary metabolites, antimicrobial peptides, phenolic compounds, etc. [50].

**Fig 6:** The antioxidant activity of *P*. *pentosaceus* OBK05. DPPH and HRS radical scavenging activities (%) using different concentration of CFS. Each value is expressed as (mean ± S.D, n = 3). MRS broth was treated as negative control and ascorbic acid as positive control. The error bars indicate a statistically significant difference at p <0.05 within each row comparing the DPPH and HRS radical scavenging activity.

### Bile salt hydrolase and cholesterol assimilation ability

Bile salt hydrolase enzyme produced by LAB liberates free amino acid and bile from conjugated bile salt. It is an indicator of cholesterol reduction by probiotic organisms and is considered an important probiotic traits. The probiotic strain OBK05 deconjugates taurodeoxycholic acid through hydrolysis and liberates free amino acid (Taurine) and bile salt (deoxycholic acid), which is represented as a zone of hydrolysis in the medium (Fig 7A and 7B). The OBK05 strain showed various levels of cholesterol removal from the growth medium incubated at different time intervals. The lowering of cholesterol in cell-free supernatant (CFS) was observed continuously at different time intervals like 12 h, 24 h and 48 h. The quantity of cholesterol reduction from the growth medium was observed to be gradually increased from 17 to 67% (Fig 7C), which is comparably higher than the previous study where the *P*. *pentosaceus* LJR5 isolated from rumen liquor of goat showed 62% reduction [38]. Similarly, a previous study [6] revealed 40% reduction in cholesterol by *P*. *pentosaceus* KID7 isolated from finger millet. These findings provide a significant design for the follow-up studies to assess cholesterol reduction ability of probiotic organisms in humans.

**Fig 7:** Bile salt hydrolase and cholesterol assimilation potential of the probiotic bacterium *P*. *pentosaceus* OBK05. (A) Un-cultured Taurodeoxycholic acid, (B) OBK05 cultured Taurodeoxycholic acid developed precipitation around the well, which indicates BSH activity, (C) Gradual increase in cholesterol reduction at 12, 24 and 48 h of incubation. Experiments were carried out in triplicates, and data with Error bars represent as the Mean ± S.D. values of the independent investigation (p <0.05).

## Conclusion

The outcome of the present study reveals that *Pediococcus pentosaceus* OBK05 strain isolated from buttermilk, possesses key *in vitro* probiotic characteristics. The probiotic strain was better able to tolerate ox bile, low pH and aggregation activities than the standard probiotic strain *L*. *acidophilus* MTCC10307. The antagonistic activity of the OBK05 strain was broader for major bacterial pathogens like *Pseudomonas aeruginosa* and *Bacillus subtilis*. Further, the OBK05 strain was found to possess nontransferable chromosomal borne resistance to significant antibiotics that restricts the horizontal gene transfer to pathogens, making them antibiotic-resistant. The probiotic strain OBK05 exhibited a higher degree of antioxidant and cholesterol-lowering activity *in vitro*. From the present study results, it can be concluded that the lactic acid bacterial isolate *Pediococcus pentosaceus* OBK05 can be used as a potential probiotic organism either in the form of powdered culture or with dairy food products. The effectiveness of this probiotic formulation represents a step ahead in the nutritional treatment of hypercholesterolemia. This organism can also be a great alternative to the conventional probiotic lactic acid bacteria, used along with strong antibiotics to treat various infections.

## Supporting information

S1 Data Suplementary data for tables. (XLSX)

S2 Data Supplementary data for figures. (XLSX)
